The article "Synthesis and Analysis of Impregnation on Activated Carbon in Multiwalled Carbon Nanotube for Cu Adsorption from Wastewater" was published in 2022. Journal: Bioinorg Chem Appl.

# Synthesis and Analysis of Impregnation on Activated Carbon in Multiwalled Carbon Nanotube for Cu Adsorption from Wastewater

**DOI:** 10.1155/2022/7470263

**Published:** 2022-07-31

**Authors:** L. Natrayan, P. V. Arul Kumar, Joshuva Arockia Dhanraj, S. Kaliappan, N. S. Sivakumar, Pravin P. Patil, S. Sekar, Prabhu Paramasivam

**Affiliations:** ^1^Department of Mechanical Engineering, Saveetha School of Engineering, SIMATS, Chennai 602105, Tamil Nadu, India; ^2^Department of Mechanical Engineering, Bharath Niketan Engineering College, Aundipatti, Theni 625531, Tamil Nadu, India; ^3^Centre for Automation and Robotics (ANRO), Department of Mechatronics Engineering, Hindustan Institute of Technology and Science, Padur, Chennai 603103, India; ^4^Department of Mechanical Engineering, Velammal Institute of Technology, Chennai 601204, Tamil Nadu, India; ^5^Department of Mechatronics Engineering, TISHK International University, Erbil, Iraq; ^6^Department of Mechanical Engineering, Graphic Era Deemed to be University, Bell Road, Clement Town 248002, Dehradun, Uttarakhand, India; ^7^Department of Mechanical Engineering, Rajalakshmi Engineering College, Rajalakshmi Nagar Thandalam, Chennai 602105, Tamil Nadu, India; ^8^Department of Mechanical Engineering, College of Engineering and Technology, Mettu University, Mettu 318, Ethiopia

## Abstract

Industrial wastes contain more toxins that get dissolved in the rivers and lakes, which are means of freshwater reservoirs. The contamination of freshwater leads to various issues for microorganisms and humans. This paper proposes a novel method to remove excess copper from the water. The nanotubes are used as a powder in membrane form to remove the copper from the water. The multiwalled carbon nanotube is widely used as a membrane for filtration. It contains many graphene layers of nm size that easily adsorbs the copper when the water permeates through it. Activated carbon is the earliest and most economical method that also adsorbs copper to a certain extent. This paper proposes the methods of involving the activated carbon in the multiwalled carbon nanotube to improve the adsorption capability of the copper. Here, activated carbon is impregnated on the multiwalled carbon nanotube's defect and imperfect surface areas. It makes more adsorption sites on the surface, increasing the adsorption amount. The same method is applied to Hydroxyl functionalized multiwalled carbon nanotubes. Both the methods showed better results and increased the copper removal. The functionalized method removed 93.82% copper, whereas the nonfunctionalized method removed 80.62% copper from the water.

## 1. Introduction

Copper plays a major role in keeping the body's immune system healthy. It also plays a major role in the formation of red blood cells. The recommended daily allowance of copper intake to the human body is 1 to 10 mg, whereas above the recommended value, it is considered toxic [1]. Both high and lower consumption of copper leads to brain diseases like Wilson's, Alzheimer, and Menkes. The deficiency of copper can be overcome by taking the proper supplements, but copper's toxicity needs to be addressed [2]. Nowadays, there is the possibility of copper toxicity in the water because of the leakage of copper from the copper pipes used in the industries which undergone corrosion [3]. It increases the level of copper higher than 6 mg/l in the water, which is hazardous to microorganisms and the human body [4]. When copper is mixed with water, it will be tasteless, odourless, and not visible. So proper testing and laboratory results are required to find the amount present in the water [5]. The extraction experiments were performed at 22°C. The results indicated that the stripping of chromium (III) from the loaded organic phase with HCl is depended on the acid strength. A contact time of 30 min yielded a maximum separation of chromium (III) was approximately 50% with up to 3 mol/L acids [6]. The separation of chromium was (90%) achieved in 29 min with mol/L acid, but this is maybe led to the decomposition of the extractant. Using HNO_3_ or H_2_SO_4_, 6 mol/L HNO_3_ yielded only 45% separation of chromium (III) in 10 min, and 10 mol/L HNO_3_ resulted in 65% separation in 20 min [7]. The maximum recovery was obtained at a pH was 4.7, and 1.0 ml HNO_3_ was used as an eluent. The higher preconcentration flow rate indicates that the efficiency of mass transport of Pb (II) ions onto MWCNTs is decreased due to the low kinetic adsorption [8]. The adsorption of Cr3+ and Cr6+, Ni2+, Cu2+, Zn2+, and Pb2+ by SPE have been studied to some extent by other authors, and it was found that the process could facilitate complex formation with the chelating agents [9]. The aqueous sample solutions contain chromium ions, the pH was maintained at 8, and the flow rate was 6.5 mL/min. The desorption of chromium using 500 *μ*L of 1M HNO_3_ was used [10].

The article "Synthesis and Analysis of Impregnation on Activated Carbon in Multiwalled Carbon Nanotube for Cu Adsorption from Wastewater" was published in 2022. Journal: Bioinorg Chem Appl.

The copper removal from water can be carried out using different methods: chemical precipitation, dissolved air floatation, adsorption, ion exchange, membrane filtration, etc. [11]. Among these techniques, the adsorption is easy and economical for copper removal. It carries out a relatively simple procedure of adsorbing the copper by the adsorbents [12]. Nanoparticles are widely used for adsorption because of their unique adsorption capacity. The preconcentration and separation were based on the chelating polymeric matrix. It is due to the presence of the vinyl pyridine-divinylbenzene resin group. The copolymer was synthesized by suspension polymerization [13]. The preconcentration and separation of Pb (II) ion based on the MWCNTs coupled online to FAAS was developed. The garlic samples were decomposed using 10 mL of concentrated HNO_3_ and 4 mL of H_2_O_2_ [14]. The following are the nanoparticles involved: carbon-based, metal NP, metal oxide-based, and nanocomposites [15]. The large surface area and porosity characteristics of the adsorbent in carbon-based materials help absorb more copper from the water, which helps better filtration [16]. Many carbon-based materials like porous carbon, activated carbon, carbon nanotubes [17], etc., are used. Carbon nanotubes are among the carbon-based materials with high tensile strength and good temperature stability, increasing the system's reliability. There are three types of nanotubes [18]: single-walled, doubly walled, and multiwalled. The multiwalled nanotubes are gaining more attention because they contain more layers of different diameters, which helps filter the contaminants of various particle sizes [19]. The major advances in the performance of SPE systems for metal ion separations could be achieved if future investigations are carried out in a more systematic and environment-friendly way [20]. Most of the studies found in the literature were carried out with synthetic solutions, and only a few studies used real effluents. It was decided to evolve a technique for separating Cr3+ and Cr6+, Ni2+, Cu2+, Cd2+, Zn2+, and Pb2+ from industrial wastewater, groundwater, and well water [21]. The main disadvantages of these processes are inherent limitations from SPE due to loading limitation, losses of metal ions in the interfacial section, organic solvents used, primary and secondary sludge generation, high cost and inconvenient operational conditions, etc., [22]. These methods are still unsatisfactory for the preconcentration and separation of heavy metals in the environmental samples [23].

In carbon-based materials, activated carbon is another economical method used for adsorption. Many research works reported that activated carbon's main disadvantage had not adsorbed lower molecular weight compounds [24]. This research aims to investigate the novel impregnation of activated carbon in the multiwalled carbon nanotubes to improve the adsorption capability of copper from the water. This paper proposes the impregnation of activated carbon and multiwalled carbon nanotubes to increase adsorption capability efficiency. The Langmuir and Freundlich isotherms are used to manipulate and analyze the newly proposed method.

The article "Synthesis and Analysis of Impregnation on Activated Carbon in Multiwalled Carbon Nanotube for Cu Adsorption from Wastewater" was published in 2022. Journal: Bioinorg Chem Appl.

## 2. Materials and Method

### 2.1. Multiwalled Carbon Nanotubes (MWCNT)

More than two layers of graphene sheet rolled up in a circular form called multiwalled carbon nanotubes. The Russian Doll model and the Parchment model are involved in forming multiwalled carbon nanotubes. The Russian Doll model will have many walls of graphene sheet rolled up in concentric circles. The Parchment model uses only a single graphene sheet to roll itself in different diameters [25]. The diameter difference between the inner walls will be 0.34 nm. The length of it will be 20 *μ*m. The angular positioning of graphene layers will be o to 90 degrees. The main properties of multiwalled carbon nanotubes are less weight, more temperature stability, corrosion resistance, and highly tensile and electrical conductivity [26]. Multiwalled carbon nanotubes are used as electrical conductors, thermal conductors, communication purposes, adsorption techniques, solar cells, batteries, nanoelectronics, energy storage, flat panel display, etc.

Many graphene layers are present in a multiwalled carbon nanotube, so there is more possibility of defects in the nanotube than single-walled nanotube. The defects are usually formed during the synthesis process [27]. The surface defects occur on the multiwalled carbon nanotube due to the imperfection in the layers. But in the multiwalled carbon nanotube, modification can occur at the last layer. The additional functionality can be obtained by adding functional groups like carboxylic groups, amides, hydroxides, etc., to improve the adsorption capability [28]. The functionalized groups of multiwalled carbon nanotubes show enhanced dispersion performances, separation of certain organic and inorganic compounds, sorting elements, and manipulation purposes. In biomedical application, the powdered form of MWCNT with the functional groups get functionalized with proteins, enzymes, nucleic acids, carbohydrates, drugs, and antibodies [29].

The COOH- multiwalled carbon nanotube can be formed by adding carboxyl groups to the nanotubes' defects, surface, and end. It is powder form and synthesized using the catalytic carbon vapour deposition method. The main application is adsorption, enhanced electric conductivity, used as an additive, biomedical applications, etc., [30]. The volumetric method usually produces the hydroxyl group of multiwalled carbon nanotubes. They have high thermal conductivity and hydrogen storing capacity. The amides-based multiwalled carbon nanotube usually has fluorescence properties according to the functionalized amide group. It produces a different fluorescence capability [31]. It uses usual chemical decomposition processes and functionalizes with amide groups. According to the adsorbate, the different functional groups are characterized and synthesized. The OH groups adsorb the organic and inorganic compounds from the water and help infiltration processes. The adsorption capability of the multiwalled carbon nanotube was improved by hydroxyl-based functionalization [32]. The multiwalled carbon nanotubes are manufactured as a membrane to remove unwanted chemicals through impregnation.

The article "Synthesis and Analysis of Impregnation on Activated Carbon in Multiwalled Carbon Nanotube for Cu Adsorption from Wastewater" was published in 2022. Journal: Bioinorg Chem Appl.

### 2.2. Activated Carbon

Activated carbon is the oldest method used to purify air and water. Activated carbons are synthesized by heating the charcoal at a high temperature with the gas. The activated carbon's large surface area absorbs the surface's impurities. The activated carbon adsorbs more carbon-based impurities, chlorine, and volatile organic compounds [33]. The various kinds of activated carbon are powdered form, impregnated form, granular form, woven carbon, polymer-coated form, etc. They are made from coconut shells, peat, petroleum-based compounds, etc. The applications include dye additives, biomedical, industries, wastewater treatment, water filtration, and air pollution treatment [34]. The main benefits of charcoal filtering are economical, maintenance easier, filter only impurities, and flavorful and healthier water [35].

## 3. Experimental Procedure

There are various methods for removing toxic ions from the water like an ionic exchange, reverse osmosis, biosorption, coagulation, extraction, etc. Adsorption is the technique widely used where the adsorbent adsorbs the adsorbate. It is a quite easier method of removal of toxic ions. Here, the toxic ions are considered the adsorbate, and adsorbents are the materials that adsorb it [36]. Usually, adsorbents are carbonaceous because when carbon reacts with toxic ions, it removes the oxide part and metal part separately. One toxic ion is copper when its amount increases in the water by more than 10 mg. Copper usually helps in the metabolic system of the human body for various functions [37]. But if their amount increases above 6 mg, it irritates the eye and mouth and produces digestion discomfort. More than 10 mg of copper in the water leads to brain disorders, psychiatric problems, kidney disorders, etc. Nowadays, more industrial waste is getting mixed up in the rivers and lakes, a new drinking water source [38]. The corrosion of the copper pipes used in the industries is the main source of more copper discharged into the water. So the removal of copper is necessary to maintain the good nutrient level of the water [39].

In the reaction of copper with water, oxygen, and carbon dioxide, the following reaction will take place:

(1) $$\begin{array}{c} 2\text{Cu}+{\text{H}}_{2}\text{O}+{\text{CO}}_{2}+{\text{O}}_{2}⟶\text{Cu}{\left(\text{OH}\right)}_{2}+{\text{CuCO}}_{3}. \end{array}$$

The byproduct of copper when it reacts with water and air is copper hydroxide and copper carbonate. The copper hydroxide produces eye irritation, and copper carbonate produces mouth irritation in the human body.

The article "Synthesis and Analysis of Impregnation on Activated Carbon in Multiwalled Carbon Nanotube for Cu Adsorption from Wastewater" was published in 2022. Journal: Bioinorg Chem Appl.

The multiwalled carbon nanotubes are highly tensile, which suits all environments. The multiwalled carbon nanotubes have different layers that easily adsorb the copper from the water [40]. The large surface area in the multiwalled carbon nanotubes permeates the copper compounds to sit on the different sites present on their surface. No reactions will occur between copper and the graphene layers in the nanotubes [41].

This paper proposes a novel method of impregnating activated carbon in the multiwalled carbon nanotubes to improve the adsorption capability of copper from the water. From the literature, it is seen that activated carbon adsorption capability is very much less compared to the other techniques present. But this paper proposes the usage of activated carbon in the defect areas sites of the surface of the multiwalled carbon nanotubes. The imperfect sites on the surface of the multiwalled carbon nanotubes reduce the adsorption rate. So, impregnating activated carbon on those sites will increase the adsorption rate [42]. The activated carbon reduces the effects of carbonaceous impurities present in the graphene sheets, which is also one of the reasons for hindering the adsorption capability. The porous size distribution will become uniform on the surface, which helps the copper adsorbed evenly on the surfaces. Due to the large surface area property of both activated carbon and the multiwalled carbon nanotube, many toxic ions can be adsorbed. There will be more ionic exchange and Vander wall's reaction on the sites [43]. Thus, the reduction in the adsorption rate due to the surface defects can be overcome by using activated carbon.

The following equation gives the reaction of copper with carbon:

(2) $$\begin{array}{c} \text{Cu}{\left(\text{OH}\right)}_{2}⟶\text{CuO}+{\text{H}}_{2}\\ {\text{CuCO}}_{3}⟶\text{CuO}+{\text{CO}}_{2}\\ 2\text{CuO}+\text{C}⟶2\text{Cu}+{\text{CO}}_{2}. \end{array}$$

The Cu (OH)_2_ and CuCO_3_ are byproducts obtained from the above three reactions when the copper reacts with water and air. When reduced, copper hydroxide and copper carbonate give the copper oxide. The copper oxide produces pure copper metal and carbon dioxide when it reacts with carbon.

In addition to the conventional multiwalled carbon nanotubes, the paper applies the above-explained concept to the Hydroxyl functionalized multiwalled carbon nanotubes. Because the Hydroxyl functionalized, multiwalled carbon nanotubes yield more adsorption capability than the conventional ones [44]. The OH groups and activated carbon are impregnated on the last layer of the multiwalled carbon nanotubes. Now there is the possibility that more sites will be present for the toxic ions to get adsorbed. There will be more surface reactions and ionic exchange [45]. At last, the copper obtained will be filtered by the inner layers of multiwalled carbon nanotubes, which act as membranes for the filtration process.

The article "Synthesis and Analysis of Impregnation on Activated Carbon in Multiwalled Carbon Nanotube for Cu Adsorption from Wastewater" was published in 2022. Journal: Bioinorg Chem Appl.

The Langmuir adsorption isotherm is used as a formula for measuring the proposed work's adsorption capacity. The following assumptions are made in the Langmuir adsorption isotherms:

- The immobile state of adsorbate should get adsorbed
- The energy is equivalent in all sites of adsorbent
- The site should have the ability to hold at least one molecule
- The surface of the adsorbent must be homogeneous
- The interaction of molecules on the adsorbent's adjacent sites should be either zero or ideal

The Langmuir adsorption isotherms formula is given in the following equation:

(3) $$\begin{array}{c} \theta_{A}=\frac{K_{\text{eq}}^{A}p^{A}}{1+K_{\text{eq}}^{A}p^{A}}, \end{array}$$

where *θ*_*A*_—fractional occupancy of adsorbent sites, *K*_eq_^*A*^—Equilibrium constant, *p*^*A*^—Adsorbate's partial pressure.

Another equation described by Langmuir is given in the following equation:

(4) $$\begin{array}{c} \theta_{A}=\frac{V}{V_{m}}, \end{array}$$

where *V*_*m*_–Volume of adsorbate in an immobile gaseous state, *V*–Volume of homogeneous adsorbent sites where the adsorbates get occupied.

Another isotherm is also used for the empirical calculation to find the adsorption capability, which is the derived method from the Langmuir isotherm is the Freundlich isotherm. This isotherm helps find the binding nature of the heterogeneous adsorbate and adsorbent materials. A comparative study is made using both the isotherms to impregnate activated carbon in the normal and Hydroxyl functionalized multi-walled carbon nanotubes. The empirical relation of Freundlich isotherm is given by the following equation:

(5) $$\begin{array}{c} \frac{x}{m}=Kp^{1/n}. \end{array}$$

*X*—adsorbate mass, *M*—adsorbent mass, *p*—equilibrium pressure, *K* and *n* are constants that depend on the adsorbate and adsorbent depending on the temperature.

## 4. Results and Discussions

The adsorption capacity is studied by adding 0.2 to 0.4 g of multiwalled nanotube content in the solution of 25–500 ml of pH ranging from 2 to 6 values.  Table 1 shows the values used for the analysis.  Table 2 shows the constant values used for the Langmuir Isotherm algorithm.  Table 3 shows the constant values used for the Freundlich Isotherm algorithm.

The article "Synthesis and Analysis of Impregnation on Activated Carbon in Multiwalled Carbon Nanotube for Cu Adsorption from Wastewater" was published in 2022. Journal: Bioinorg Chem Appl.

Figure 1 shows the plot of isotherm calculated to obtain the analysis of activated carbon on the multiwalled carbon nanotube. At the pressure of 77 K, the activated carbon is settled at the imperfection areas of the multiwalled carbon nanotube. This graph is plotted to study the interaction between activated and multiwalled carbon nanotubes. Here, the activated carbon is attached by the physisorption method [46]. This attached activated carbon has large pores, which increases the absorption rate of the copper from the water. It is seen that the volume of activated carbon increases with an increase in the ratio of adsorbate to the adsorbent material. Here we considered the even distribution of activated carbon on the multiwalled carbon nanotube for simulation purposes. The activated carbon mostly gets impregnated in the imperfect or defective areas rather than in normal surface areas. Only the upper layers of the multiwalled carbon nanotube are subjected to the impregnation of the activated carbon [47]. Activated carbon adsorbs the ionic elements by either ionic reaction or Vander Wal forces. If the ionic element is present in oxide form, the reaction will result in that particular element and carbon dioxide. So it will be easy for the multi-walled carbon nanotube to filter the ions because the membrane form will disperse the molecular size of the ion.

Figure 2 shows the copper removal vs time. The comparison of activated carbon with multiwalled carbon nanotube and activated carbon with Hydroxyl multiwalled carbon nanotube is made. The Hydroxyl functionalized form of the proposed method yields good results compared to the normal multiwalled carbon nanotube [48]. After 40 minutes, both methods reach the saturation point where copper removal maintains the same level. So from the result, it is seen that the water has utmost of 34.9% of copper, which Hydroxyl adsorbs functionalized multiwalled carbon nanotube and 29.89% of copper is adsorbed by normal method [49]. The Hydroxyl functionalized multiwalled carbon nanotube impregnated with activated carbon attains 14.3% efficiency compared to the multiwalled carbon nanotube impregnated with activated carbon nanotube. The pH value is considered to be random, between 2 and 6. From the graph, it is seen that the copper removal percentage increases with time. The ionic exchange takes place between the activated carbon and the copper oxide. More the time the reaction occurs, the nanotube starts to disperse the copper through the membrane within which filtering takes place [50]. There is the possibility that many toxic compounds are also adsorbed, but the process mainly concentrates on the copper adsorption of the nanotubes. If the nanotubes adsorb more copper from the water, it depletes the nutrient value of the water.

The article "Synthesis and Analysis of Impregnation on Activated Carbon in Multiwalled Carbon Nanotube for Cu Adsorption from Wastewater" was published in 2022. Journal: Bioinorg Chem Appl.

In Figure 3, the plot of ionic strength vs adsorption percentage is done. As the paper discussed earlier regarding Figure 2, more ion exchange will occur as time takes. More chemical reactions will also happen. So there will be more adsorption of copper is carried out both by activated carbon and multi-walled carbon nanotube. The added hydroxyl groups also react with the copper and increase its removal [51]. The adsorption percentage is measured after 20 minutes because the active reactions occur after that particular period. From Figure 3, it is clear that as the ionic strength, the adsorption percentage also increases. But it takes some time for the ionic reaction; after reaching the ionic strength of 35.5 mg/l of copper, only the adsorption percentage rises. As discussed above, the Hydroxyl functionalized multiwalled carbon nanotube impregnated with activated carbon nanotube shows more adsorption percentage than the normal one [52]. The Hydroxyl functionalized multiwalled carbon nanotube impregnated with activated carbon shows a comparatively 13.2% more adsorption percentage.

Figure 4 shows the Freundlich isotherm plot.  Table 3 shows the value of constants used for empirical calculation of the proposed works. The isotherm is applied for both methods. The logarithmic scale measures the amount of adsorbate mass adsorbed from the concentration taken in 50 ml of solution. The *K* and *n* values are obtained, particularly considering the copper element alone [53]. But this is practically quite impossible. The Hydroxyl functionalized multiwalled nanotube shows more adsorption mass from the amount of solution taken at given pressure and temperature. Usually, 77 K pressure is considered when calculating the empirical values. The logarithmic scale is chosen, which helps to bring the values in a good straight line. In this isotherm, the adsorbate and adsorbent may be any form but should react at the given temperature and pressure [54].

Figure 5 shows the Langmuir isotherm plot for the proposed work.  Table 2 shows the constants used for manipulation. The constants are taken according to the mass value of the copper. The Langmuir isotherm considers the even distribution of the surface adsorbent used [55]. Here, the paper uses activated carbon and hydroxyl groups on the multiwalled carbon nanotube to overcome the imperfection and improve the adsorption ability of ions. The hydroxyl-based work shows better interaction between adsorbate and adsorbent than the normal multiwalled carbon nanotube with activated carbon.

The article "Synthesis and Analysis of Impregnation on Activated Carbon in Multiwalled Carbon Nanotube for Cu Adsorption from Wastewater" was published in 2022. Journal: Bioinorg Chem Appl.

## 5. Conclusion

The proposed work efficiency is manipulated using different algorithms and different parameters. The following conclusion has been drawn:

- The method with and without Hydroxyl functionalized carbon nanotube impregnated with activated carbon shows better adsorption capability. But the Hydroxyl functionalized method yields a better result of 93.82% adsorption efficiency and 34.59% copper removal from 50 mL of water containing a 2–6 pH value.
- The nonfunctionalized multiwalled carbon nanotube impregnated with activated carbon yields an 80.69% adsorption percentage and 29.69% copper removed from the water.
- The Langmuir and Freundlich others were calculated, providing better interaction between the copper adsorbates and the proposed model of multiwalled carbon nanotube.
- The calculation for the amount of activated carbon impregnated on the surface of the multiwalled carbon nanotube was also done. A comparative study was made where the functionalized proposed work method yields better results than the nonfunctionalized multiwalled carbon nanotube.

The proposed methodology is quite complex, but it is also very economical. The further scope of this work can be carried out by characterizing the nanotubes' surface area, which helps to improve adsorption capability still more.

## Figures and Tables

**Figure 1:** Isotherm at 77 K.

**Figure 2:** Cu removal vs time.

**Figure 3:** Ionic strength vs adsorption percentage.

**Figure 4:** Freundlich model plot.

**Figure 5:** Langmuir model plot.

**Table 1:** Parameters for analysis.

Parameters	Values
pH	2–6
Nanotube amount	0.2–0.6 g
Sample volume	25–500 ml
Certified Cu value	17.3 ± 1.0 *μ*g/g

**Table 2:** Langmuir isotherm constant values.

Langmuir Isotherm Constants	*K*_eq_^*A*^	*R*_*L*_	*R* ^2^
	0.463 l/mg	0.041	0.997

**Table 3:** Freundlich isotherm constant values.

Freundlich Isotherm Constants	*K*	*N*	*R* ^2^
	4.071	3.300	0.929

## Data Availability

The data used to support the findings of this study are included within the article.
